The article "Construction of Home Product Design System Based on Self-Encoder Depth Neural Network" was published in 2022. Journal: Comput Intell Neurosci.

# Construction of Home Product Design System Based on Self-Encoder Depth Neural Network

**DOI:** 10.1155/2022/8331504

**Published:** 2022-04-21

**Authors:** Guangpu Lu

**Affiliations:** School of Art, Huzhou University, Huzhou, Zhejiang 313000, China

## Abstract

The traditional home product design system mainly depends on relatively shallow learning network, relatively simple embedded technology and Internet of things technology. The traditional home design system mainly depends on the traditional self-encoder technology. When combined with the deep neural network, this technology has serious defects in the computer vision algorithm, resulting in the serious waste of the corresponding system storage and computing resources, the corresponding system learning efficiency is relatively poor and the learning ability is weak. Based on this, this paper will build a home product design system based on the deep neural network of self-encoder. By improving the sparsity of self-encoder in the process of learning and training, we can further improve the sparsity of the system and further optimize the structure of self-encoder in the design system, The performance of the deep learning model of the design system is further improved through the hierarchical features continuously learned by the self-encoder in the process of home case design. Based on the optimization of the home product design system in this paper, the system effectively improves and improves the accuracy and stability of the internal feature classifier of the system, and improves the overall performance of the furniture design system. In the specific system construction part, based on ZigBee technology and embedded technology as the design carrier, and adhering to the goal of simplicity, intelligence and convenience, this paper designs and constructs the home product design system. The experimental results show that the noise processing level of the proposed home product design system is lower than 4-5db compared with the traditional design system, and the corresponding image classification accuracy is about 4% higher than the traditional design system. Therefore, the experimental results show that the home design system proposed in this paper has obvious advantages.

## 1. Introduction

With the continuous development of embedded technology, Internet of things technology and other related technologies, home product design system is also changing. A complete home product design system includes the integration of embedded theory, server construction and application technology, computer control and design technology, single chip microcomputer principle and control technology, wireless communication technology and other technologies [1–3]. However, the current traditional home product design system relies too much on simple embedded system and Internet of things system, and its research on its intelligence is very limited. As a result, the home product design system cannot meet the actual needs of designers and users [4, 5]. At the same time, the products designed by the current home design system also have the problems of single product structure, serious functional homogeneity, intelligent service and low degree of adaptability [6]. Based on this, a large number of companies and researchers have invested a lot of time and energy to study the home product design system, and attempt to establish a personalized, intelligent, personalized and simplified design system, in order to meet the needs of designers and customers.

The article "Construction of Home Product Design System Based on Self-Encoder Depth Neural Network" was published in 2022. Journal: Comput Intell Neurosci.

As a rapidly developing learning algorithm in recent years, deep neural network based on self-encoder has been widely studied and applied in the fields of multimedia, intelligent design, speech control, image and video analysis and computer vision [7]. Among them, neural network model is extremely important for deep neural network. At present, its main development directions are divided into four types, corresponding to cyclic neural network, long-term and short-term memory neural network, convolution neural network and residual neural network [8–10]. The continuous development of deep neural network technology based on self-encoder also promotes the rapid development of home product design system. In home design system, deep neural network technology based on self-encoder focuses on improving home image processing performance and solving various complex images, signals and requirements, at the same time, the application of self-encoder technology can solve the learning problems of input data and the disadvantages of deep neural network at the model training level [11–13]. At the level of deep neural network training, a large number of researchers have also studied. Its mainstream algorithm mainly focuses on the research of back-propagation algorithm, and the core of back-propagation algorithm mainly focuses on the optimization of objective function. The algorithm points out that although deep neural network algorithm has strong representation ability, this algorithm can also solve the problem of poor generalization ability of traditional algorithms; As for the poor generalization ability of traditional neural networks, relevant researchers pointed out that it is mainly reflected in the serious lack of label training data, which will lead to the phenomenon of over fitting of the model; The corresponding local extremum problem is mainly reflected in the non-concave optimization problem. This problem is mainly reflected in the existence of a large number of poor local extremum points in the space. Once based on the traditional neural algorithm, the search will enter an extremely bad extremum point and fall into a dead cycle; Corresponding gradient dispersion problem. In the traditional neural network system, once the algorithm based on correlation gradient is optimized, the initial grass-roots weight transformation will become extremely slow, so that it cannot learn effectively from the samples. At present, the research of deep neural network technology based on self-encoder in household product design system is still deepening, and the corresponding technology is also developing. At the level of home product design system, the traditional home design is only limited to “imitation design” and “batch design”, which ignores the personalization, intelligence and self-learning of design. Based on this part, researchers and designers optimize and improve it. Relevant European and American researchers focused on introducing the concepts of intelligence and ecology into home product design, analysed and optimized it based on this, and achieved certain results; Some Korean designers have introduced Internet of things technology into home product design, which makes home design more intelligent and scientific.

The article "Construction of Home Product Design System Based on Self-Encoder Depth Neural Network" was published in 2022. Journal: Comput Intell Neurosci.

Based on the above analysis of the current research status of home product design system and self-encoder deep neural network technology, this paper will conduct in-depth research based on this status, and strive to solve the improvement and optimization problem of home product design system based on self-encoder deep neural network technology. Based on this, this paper will build a home product design system based on the deep neural network of self -encoder. By improving the sparsity of self-encoder in the process of learning and training, we can further improve the sparsity of the system and further optimize the structure of self-encoder in the design system, the performance of the deep learning model of the design system is further improved through the hierarchical features continuously learned by the self-encoder in the process of home case design. Based on the optimization of the home product design system in this paper, the system effectively improves and improves the accuracy and stability of the internal feature classifier of the system, and improves the overall performance of the furniture design system. In the specific system construction part, based on ZigBee technology [14–17] and embedded technology as the design carrier, and adhering to the goal of simplicity, intelligence and convenience, this paper designs and constructs the home product design system. The experimental results show that the system proposed in this paper has a qualitative leap compared with the traditional design system.

The article "Construction of Home Product Design System Based on Self-Encoder Depth Neural Network" was published in 2022. Journal: Comput Intell Neurosci.

The structure of this paper is as follows: in the second section, this paper will focus on the current research status of home product design system based on self-encoder depth neural network, and specifically analyse the development status and technical implementation of self-encoder depth neural network technology; The third section of this paper will analyse the technology of home product design system based on self-encoder depth neural network, focus on the optimization technology based on self-encoder depth neural network, and give the construction scheme of home product design system; The fourth section of this paper will verify the household product design system designed in this paper, analyse the experimental data and draw the corresponding conclusions; Finally, this paper will be summarized.

## 2. Related Research and Analysis: Analysis of the Current Situation of Home Product Design System Based on Self-Encoder Depth Neural Network

At present, the research and analysis of home product design system based on self-encoder deep neural network mainly focuses on the technical level and demand level [18–20]. At the corresponding technical level, the mainstream research is mainly the research of deep neural network technology based on self-encoder, which is mainly committed to solving the problems of sparsity, recognition accuracy and stability [14, 21, 22]. Relevant researchers in Europe and America have proposed the auxiliary greedy algorithm of neural network, which is only an important practical argument for the fusion of deep neural network and self -encoder. At the same time, the experimental results of the algorithm also show that the training efficiency of the model has been greatly improved [23–26]; In order to solve the problem of depth neural network in image recognition accuracy, German research institutions and relevant researchers pointed out that considering the sparsity feature into depth neural network is conducive to improving the image classification performance of the system [27]; In terms of corresponding algorithm efficiency, relevant researchers in the United States proposed to use the nonlinear coding function of soft threshold operator to predict sparse coding [28]. At the research level of deep neural network image denoising, a large number of researchers have used a variety of different technologies for research and analysis. Relevant Chinese researchers have proposed an optimized transformation algorithm to solve the “surround” problem, which is mainly based on the combination of hard threshold denoising technology and sub-band related image denoising algorithm, thus, the retention and thinning of image edge features are realized, which further improves the performance of self-encoder depth neural network technology [29, 30]; Relevant Japanese researchers gradually threshold denoising algorithm, which mainly establishes the corresponding mathematical model for each sub block through generalized normal distribution, and adopts sparse representation algorithm for specific images [31].

The article "Construction of Home Product Design System Based on Self-Encoder Depth Neural Network" was published in 2022. Journal: Comput Intell Neurosci.

## 3. Optimization and Construction of Home Product Design System Based on Self-Encoder Depth Neural Network

In this section, the optimization of home product design system based on self-encoder deep neural network will be analysed and studied. As shown in Figure 1, the optimization framework of home product design system under this concept is shown. From the figure, it can be seen that the design system includes five levels of content, corresponding to: Home Product wireless node part, home product supporting intelligent gateway part, Embedded server part, user operating system part and deep neural network algorithm part based on self-encoder. The configuration level of the whole system mainly includes the design of hardware and software, in which the design of hardware mainly includes the design of various sensor modules, storage modules, communication modules and power supply modules. The corresponding wireless node mainly includes product switch control, product sensor, intelligent data acquisition part and sensing part, and the algorithm part is mainly used to realize the optimization of deep neural network technology based on self-encoder. In terms of wireless transmission hardware, it is mainly based on ZigBee technology, and its corresponding hardware modules include wireless hardware core module, temperature acquisition module, light intensity acquisition module, switch control module, human body sensing module, gas acquisition module, etc. The corresponding software technology of wireless ZigBee mainly includes the establishment of network and the sending and receiving of wireless data. The corresponding gateway design level mainly includes the function of home main controller, data conversion function, data server function and corresponding router function. The corresponding software level mainly includes the construction of environment, the compilation and configuration of system and the connection with ZigBee wireless transmission network. At the corresponding software level, it mainly includes the optimization technology of deep neural network technology based on self-encoder and the design of web service program. The detailed description of the web-based coder technology is included in the detailed description of the web-based service program design. At the corresponding client design level, five functions are mainly considered, which are respectively: display and control of sensor node data, display of system alarm function, statistics and analysis of temperature transformation curve, whether it supports network connection gateway and serial port connection operation. At the corresponding communication protocol level, the main design content includes four levels: the consistency of system communication data, the simplification of system communication data, the security of system communication data and the scalability of system communication data. The selection of main hardware devices is also mainly based on mature hardware on the market. The hardware chips mainly involved include CC2530 minimum system, DS18B20 temperature sensor chip, etc.

The article "Construction of Home Product Design System Based on Self-Encoder Depth Neural Network" was published in 2022. Journal: Comput Intell Neurosci.

## 4. Optimization of Home Product Design System Based on Self-Encoder Depth Neural Network

This section mainly discusses how to further improve the sparsity of the system by improving the sparsity of the self-encoder in the learning and training process, and further optimize the structure of the self-encoder in the design system, so as to realize the stability of the home design system.

Based on this, this paper proposes a constraint learning method based on sparse self-encoder, and makes full use of its corresponding multi-level features for optimization.  Figure 2 shows the multi-level sparse self-encoder constraint learning algorithm used in this paper. It can be seen from the figure that the corresponding input data is the original image data, and each layer of the corresponding system is distributed with a different number of sparse self-encoders, which are mainly used to provide energy to the next layer. The corresponding nodes in the corresponding algorithm network model are adjustable, it can achieve the best parameter configuration through continuous verification in training.

Based on the above algorithm framework, Figure 3 shows the specific algorithm operation strategy. The corresponding ellipses in the figure are input and output, the corresponding diamond represents the specific operation of the system algorithm, and the corresponding symmetrical trapezoid represents the corresponding sparse self-encoder. It can be seen from the figure that the model selected in this paper is different from the traditional model and is implemented by serialization cascade, which plays an obvious role in improving the performance of individual weak learners in the system and the efficiency of the whole constraint learning algorithm. It can be seen from the figure that the classifier of the latter layer of the system takes the output of the previous layer as the input, so as to further deepen the network level and obtain a higher-level feature representation of the original input data. Multiple sparse feature representations of the original input data can be obtained through multiple cascade operations of the self-encoder, which mainly comes from the output of the encoding stages of different self-encoders at different levels. The specific operation steps are as follows:

Step 1: a sparse self-encoder is trained in advance, and the number of output neurons of the encoder is *n*. at this time, it is assumed that the input sample of the original data is *x*, the weight matrix responsible for connecting the input layer and the hidden layer is *w*, the corresponding offset vector is designed as *B*, and the corresponding activation function is designed as *f*, at this time, the eigenvector calculation formula obtained from the encoder input layer can be calculated, as shown in formula (1):
  (1) $$\begin{array}{c} f^{\left(2\right)}=B_{\left(w^{2}-W^{1}\right)*\left(x*W^{\left(2\right)}+B^{\left(2\right)}\right)}. \end{array}$$
Step 2: take the corresponding function in Step 1 as the input of the second sparse self-encoder, and further train to obtain the output of the second sparse matrix self-encoding stage. The calculation formula of the corresponding second self-encoder is shown in formula (2):
  (2) $$\begin{array}{c} f^{\left(t+1\right)}=B_{\left(w^{t+1}-W\right)*\left(x*W^{\left(t+1\right)}+B^{\left(t+1\right)}\right)}. \end{array}$$
Step 3: according to the process of Step 2, the feature attributes trained in the previous encoder are continuously transferred to the next self-encoder along the cascaded sparse self-encoder network to achieve the purpose of continuous training. The calculation formula of the feature vector obtained by the corresponding self-encoder input layer is shown in formula (3):
  (3) $$\begin{array}{c} f^{\left(t\right)}=B_{\left(w^{t}-W^{t-1}\right)*\left(x*W^{\left(t\right)}+B^{\left(t\right)}\right)}. \end{array}$$
Step 4: vertically, it is necessary to train the feature attributes of the coding stage respectively, so as to obtain the classifier model of each self-encoder and the corresponding optimal parameters of the corresponding classifier.

After completing the above learner training, we need to formulate a reasonable sparse self-encoder constraint rule. The rule used in this paper is Bayesian criterion. When using this criterion, we need to assume that each learner in the system is in an independent state. Bayesian criterion mainly includes maximum rule, minimum rule and average rule. The corresponding maximum rule selects the maximum prediction probability value of the learner, the corresponding minimum rule selects the base classifier with the minimum output probability among all the base learners, and the corresponding average rule calculates the corresponding average probability for all the base learners.

The article "Construction of Home Product Design System Based on Self-Encoder Depth Neural Network" was published in 2022. Journal: Comput Intell Neurosci.

In order to solve the corresponding image denoising problem in the home product design system, this paper designs a sparse induced self-encoder for processing. The design algorithm of the corresponding sparse induced self-encoder is shown in Figure 4. As can be seen from Figure 4, the layer by layer greedy algorithm is mainly used to continuously optimize the weight matrix between different layers. Based on this, the number of neurons in each corresponding layer is continuously reduced. On the corresponding sparse induction layer, the number of neurons can be further obtained by forcibly setting the neurons with low activation value of this layer to zero, then continuously strengthen the extraction of abstract things. Through the design of sparse induced self-encoder in this paper, the correlation between attributes can be further removed, so as to realize the continuous compression of input signal space.

In order to further reflect the difference between the sparse induced self-encoder proposed in this paper and the traditional encoder, as shown in Figure 5, the corresponding comparison frame diagram is given. From the figure, it can be seen that in the coding stage of the corresponding left model, it compresses the input original signal, but it does not do any special processing on the sparse characteristics of the original signal, The sparse induced self-encoder on the right side of the corresponding figure will further impose sparsity constraints on the basis of the coding stage, so as to obtain the more essential characteristics of the input data. In essence, the special processing corresponding to the sparse induced self-encoder is to set a certain threshold in advance, so that when the activation output value of some neurons in the feature output is lower than the threshold, the output value transmitted to the next layer is forced to be set to zero, so as to retain the neurons whose activation value is significantly higher than the threshold to a great extent, and then reduce the cardinality of the model parameters, It reduces the complexity of the system model and improves the generalization and compatibility of the system model.

## 5. Construction of Home Product Design System Based on Self-Encoder Depth Neural Network

Based on the above principle analysis, this section constructs the software and hardware of the system. The design system proposed in this paper is more inclined to the construction of software level. The corresponding hardware level mainly includes the selection of wireless transmission technology, the selection of smart home gateway and the selection of various sensors. At the corresponding software design level, it is mainly the application of deep neural network technology based on self-encoder. Based on this, the main technical framework is shown in Figure 6:

In terms of wireless transmission hardware, it is mainly based on ZigBee technology, and its corresponding hardware modules include wireless hardware core module, temperature acquisition module, light intensity acquisition module, switch control module, human body sensing module, gas acquisition module, etc. The corresponding software technology of wireless ZigBee mainly includes the establishment of network and the sending and receiving of wireless data.

The article "Construction of Home Product Design System Based on Self-Encoder Depth Neural Network" was published in 2022. Journal: Comput Intell Neurosci.

The corresponding gateway design level mainly includes the function of home main controller, data conversion function, data server function and corresponding router function. The corresponding software level mainly includes the construction of environment, the compilation and configuration of system and the connection with ZigBee wireless transmission network. The construction of development environment mainly includes the installation of virtual machine and operating system; When compiling the system, it mainly includes installing the corresponding tools and libraries, installing the corresponding git tools and installing the corresponding library files; When downloading the source code, first establish the corresponding folder and download online at the same time. After downloading, update the extension library files and corresponding software in time; When configuring the system, first configure the corresponding IP address, then configure the web interface supported by the system, then configure the SSH function of the system, finally configure the serial port of the system, and set the corresponding parameters. At the connection level between the corresponding gateway and ZigBee wireless transmission network, the network topology mainly adopts the star structure, that is, it is composed of one ZigBee coordinator and multiple ZigBee nodes, in which the corresponding ZigBee coordinator is mainly a transfer station. In this connection, the corresponding data is mainly transmitted through wired mode. In terms of expanding functions, the gateway mainly includes serial port application technology, USB port application technology and interface conversion application technology. The corresponding serial port application technology is mainly based on the hardware with serial port protocol, the corresponding USB port application technology is mainly based on the hardware level such as USB hard disk, and the interface conversion application is mainly processed based on hardware devices such as ethernet interface.

The article "Construction of Home Product Design System Based on Self-Encoder Depth Neural Network" was published in 2022. Journal: Comput Intell Neurosci.

At the corresponding software level, it mainly includes the optimization technology of deep neural network technology based on self-encoder and the design of web service program. The detailed description of the web-based coder technology is included in the detailed description of the web-based service program design.

At the corresponding client design level, five functions are mainly considered, which are respectively: display and control of sensor node data, display of system alarm function, statistics and analysis of temperature transformation curve, whether it supports network connection gateway and serial port connection operation. At the design level of the user's mobile phone client, it is mainly designed based on the open source system. In the actual design, the design language mainly used in this paper is Java. At the corresponding computer end, this paper mainly carries out the corresponding function development based on VC++. In the corresponding network application part, it mainly adopts Winsock API for development, at the same time, call the serial port software to realize the operation of serial port communication.

At the corresponding communication protocol level, the main design content includes four levels: the consistency of system communication data, the simplification of system communication data, the security of system communication data and the scalability of system communication data. The consistency of system communication data mainly refers to that all data packets should have a unified form of packet header and packet tail; The simplification of the corresponding system communication data mainly requires that the system should strictly control the bytes when designing the communication protocol level; The security of corresponding system communication data mainly refers to that the system should have specific format and identifier in the corresponding data header and data tail; The scalability of system communication data mainly refers to that the data corresponding to this paper also has strong scalability, which is convenient for the upgrading of future protocols and the addition of new functions.

## 6. Experiment and Data Analysis

In order to further verify the advantages of the home product design system based on self-encoder depth neural network proposed in this paper, this paper will take the way of indirect verification to compare its advantages with the traditional design system. The same household environment is designed with the same indicators, and the sensitivity of its environmental action is tested by detecting the gas concentration. The corresponding test equipment is the test equipment for household gas concentration test. The specific test structure is shown in Figure 7. The corresponding test steps based on Figure 7 are as follows:

  Step 1: record and record the corresponding gas concentration of the gas concentration alarm in the environment under the two environments when it is in normal operation.
  Step 2: release certain gas artificially, so that the ambient gas concentration gradually exceeds the threshold, record the gas concentration, and record the reaction time and action time of the gas concentration alarm.
  Step 3: analyse the comparative data and draw corresponding conclusions.

The article "Construction of Home Product Design System Based on Self-Encoder Depth Neural Network" was published in 2022. Journal: Comput Intell Neurosci.

According to the above experimental conditions, sort out the corresponding gas concentration test curve, as shown in Figure 8. From Figure 8, it can be seen that the designed environment of the home product design system based on self-encoder deep neural network proposed in this paper is more sensitive to relevant factors and has higher monitoring stability.

In order to verify the difference between the sparse induced self-encoder proposed in this paper and the traditional encoder, it is compared with the traditional sparse self-encoder. The main experimental object is the image in the environment, and the corresponding processed PSNR value is mainly analysed and evaluated. The corresponding experimental results are shown in Figure 9. The sparse induced self-encoder proposed in this paper has obvious performance advantages compared with other self-encoders.

In order to verify the advantages of the constraint learning method based on sparse self-encoder, the core algorithm in this paper is compared with its algorithm. The corresponding experimental results are shown in Figure 10, which can be seen from Figure 10, The algorithm proposed in this paper improves the recognition accuracy by at least 3 percentage points compared with the traditional algorithm under three constraint criteria (i.e. minimum criterion, maximum criterion and average criterion), and the stability under the corresponding average criterion is the most obvious. The experimental results further show that the constraint learning method based on sparse self-encoder proposed in this paper not only has the advantages of accuracy and feasibility in theory, but also has practical advantages in the corresponding real classified image scene.

The article "Construction of Home Product Design System Based on Self-Encoder Depth Neural Network" was published in 2022. Journal: Comput Intell Neurosci.

Based on the above analysis and related experiments, it is further verified that the home product design system based on self-encoder depth neural network proposed in this paper has not only theoretical advantages, but also corresponding advantages in practical application.

## 7. Conclusion

This paper mainly discusses and analyses the current situation, existing problems, solution and optimization of home product design system based on self-encoder depth neural network. In order to further realize the humanized, intelligent, personalized and simplified construction of the home product design system, this paper improves the sparsity of the self-encoder in the learning and training process, further improves the sparsity of the system, and further optimizes the structure of the self-encoder in the system, the performance of the deep learning model of the design system is further improved by the hierarchical features continuously learned by the self-encoder in the process of home case design. In order to verify the superiority of the system designed in this paper, based on ZigBee technology and embedded technology as the design carrier, and adhering to the goal of simplicity, intelligence and convenience, this paper designs and constructs the home product design system. The experimental results show that the system proposed in this paper has a qualitative leap compared with the traditional design system. However, there are still some remaining problems in the content of this paper, which need to be further analysed. In the follow-up research, this paper will focus on the efficiency of the algorithm and the intelligence of model learning. At the same time, this paper will further expand the application fields of the algorithm, such as video surveillance, other product design, security and so on.

## Figures and Tables

**Figure 1:** Structural block diagram of home product design system based on self-encoder depth neural network.

**Figure 2:** Framework of multi-level sparse self-encoder constrained learning algorithm.

**Figure 3:** Operation strategy diagram of multi-level sparse self-encoder constraint learning algorithm.

**Figure 4:** Design algorithm framework of sparse induced self-encoder.

**Figure 5:** Comparison block diagram of sparse induced self-encoder and traditional encoder.

**Figure 6:** Software and hardware framework of home product design system based on self-encoder deep neural network.

**Figure 7:** Test structure diagram of home product design system based on self-encoder deep neural network.

**Figure 8:** Comparison broken line block diagram.

**Figure 9:** Performance comparison curve of sparse induced self-encoder and traditional encoder under different image noise levels (a-d different image noise levels).

The article "Construction of Home Product Design System Based on Self-Encoder Depth Neural Network" was published in 2022. Journal: Comput Intell Neurosci.

**Figure 10:** Comparison curve of accuracy of different image classification algorithms under three different constraint criteria.

## Data Availability

The data used to support the findings of this study are available from the corresponding author upon request.
